# Association between Tumor Prognosis Marker Visfatin and Proinflammatory Cytokines in Hypertensive Patients

This article has been retracted.

**DOI:** 10.1155/2021/8568926

**Published:** 2021-03-16

**Authors:** Ramya Parimelazhagan, Dhamodharan Umapathy, Inmozhi Ramu Sivakamasundari, Subramaniam Sethupathy, Daoud Ali, Ramkumar Kunka Mohanram, Nalini Namasivayan

**Affiliations:** ^1^Department of Biochemistry, Faculty of Medicine, Rajah Muthiah Medical College and Hospital (RMMCH), Annamalai University, Annamalainagar 608002, India; ^2^Department of Pharmacology, Saveetha Dental College and Hospitals, Saveetha Institute of Medical and Technical Sciences, Chennai 600 077, India; ^3^Department of Zoology, College of Science King Saud University, P.O. Box 2455, Riyadh 11451, Saudi Arabia; ^4^SRM Research Institute, SRM Institute of Science and Technology, Kattankulathur 603203, India; ^5^Department of Biochemistry and Biotechnology, Faculty of Science, Annamalai University, Annamalainagar 608002, India

## Abstract

Visfatin has been reported as a risk factor and a potential diagnostic marker in cancer. It is an adipokine, secreted by visceral fat and associated with the pathogenesis of arterial hypertension. We investigated the circulatory levels of visfatin in hypertensive patients with hypertriglyceridemia, which are the risk factors for various cancers and its association with proinflammatory cytokines. A total of 81 (male/female: 33/48) subjects with or without hypertension were enrolled for this study. Group 1 was normotensive, Group 2 hypertensive, and Group 3 with hypertension with hypertriglyceridemia. Data on anthropometric and biochemical data were recorded. Plasma visfatin levels were measured using an ELISA kit. The plasma inflammatory cytokines were estimated using a multiplex bead-based assay. The results revealed that the hypertension with hypertriglyceridemia group has the highest levels of visfatin compared to the hypertension and control groups with a significant difference (*p* < 0.001). Besides, circulatory visfatin showed the strongest possible correlation with proinflammatory cytokines among hypertensive patients with hypertriglyceridemia. We found a positive correlation between visfatin and diastolic blood pressure as well as high-density lipoproteins. In conclusion, the outcomes of the present study demonstrate that plasma visfatin levels were found to be elevated in hypertensive patients with hypertriglyceridemia and associated with proinflammatory cytokines. Since hypertension has been documented as the most common comorbidity observed in cancer patients, visfatin may be a novel potential therapeutic target for hypertension in cancer patients and survivors.

## 1. Introduction

Hypertension and associated disorders affect more than one-third of the adult population worldwide [1]. Uncontrolled hypertension leads to an array of cardiovascular diseases leading to considerable morbidity and mortality. Hypertension research has progressed extensively, but the exact mechanism of blood pressure elevation is yet to be unraveled [2]. Hypertension has been documented as the most common comorbidity encountered in cancer patients [3].

Mononuclear phagocytes infiltrate the heart, the vasculature, and the kidneys during hypertension [4]. These infiltrating macrophages and T-lymphocytes secrete or induce several inflammatory cytokines [5, 6]. Particularly T-lymphocytes show a substantial role in the etiology of increased blood pressure [7]. Therapy aimed at inhibiting lymphocyte proliferation in autoimmune diseases associated with hypertension revealed a significant decrease in blood pressure. These results reinforce the theory that the immune system plays a significant role in blood pressure regulation [4, 8].

Visfatin, also named nicotinamide phosphoribosyl transferase (NAMPT), is a 52 kDa protein secreted by adipose tissue, leukocytes, hepatocytes, and muscles [9]. It has been identified as a new proinflammatory adipocytokine, which induces the monocytes and dose-dependently increases the synthesis of cytokines [10]. The anti- and proinflammatory cytokines secreted by monocytes have a considerable role in various infections/inflammatory conditions [11]. Gunes et al. reported that visfatin is associated with inflammation and endothelial dysfunction in patients with hypertension [12].

There is an increase in serum visfatin concentration during obesity, which in turn is associated with vascular inflammation and insulin resistance [13]. Enhanced visfatin levels progress cell-mediated inflammation leading to macrophage survival via IL-6 release inhibiting neutrophil apoptosis and sepsis [14]. Increased visfatin was not only observed in hypertension but also reported to increase the risk of obesity-related malignancies such as breast, endometrial, and colorectal cancer in females, whereas oral squamous cell carcinoma and gastric and bladder cancer in males [15]. The proinflammatory transcription factors such as NF-*κ*B, MAPKs, and PI3K and ROS pathways are triggered due to increased visfatin levels [16].

The increased circulating serum visfatin leads to lymph node infiltration in advanced stages of several cancers [17–19]. A state of chronic low-grade subclinical inflammation connecting to obesity is directly implicated to malignancies in hypertensive subjects with hyperlipidemic conditions [20]. Therefore, we investigated the levels of circulatory visfatin in hypertensive patients with hypertriglyceridemia, which are the risk factor for obesity-associated malignancies, and its correlations with other traditional clinical parameters and a panel of circulatory proinflammatory cytokines.

## 2. Materials and Methods

### 2.1. Study Design

This cross-sectional study was conducted in Southern India at the Rajah Muthiah Medical College, Annamalai University. A total of 81 participants consisting of 48 females and 33 males, having an average age of 52 ± 10.7 years, were evaluated in this study from November 2016 to April 2017. The study protocol was permitted by the Annamalai University ethics committee (IHEC/0189/2017). Subjects with hypertension were diagnosed based on World Health Organization criteria. A consent form was collected from all the study subjects after explaining the study objectives and benefits. The study subjects were divided into the following: group 1 were normotensive subjects (*n* = 20), group 2 were hypertensive subjects (*n* = 26), and group 3 were subjects with both hypertension and hypertriglyceridemia (*n* = 35).

### 2.2. Inclusion and Exclusion Criteria

Adult hypertensive patients under treatment with antihypertensive drugs (ACE inhibitors, angiotensin receptor blockers, and/or calcium blockers) were included in the study. Patients with a history of chronic infections, malignancy, hyper/hypothyroidism, kidney diseases, and autoimmune diseases were excluded from the study.

### 2.3. Diagnosis of Hypertension, Hypertriglyceridemia, and T2DM

The blood pressure of the study subjects was recorded using an electronic sphygmomanometer (Omron HEM-7080 and HEM-7080IT-E; Omron Corporation, Tokyo, Japan). Two separate blood pressure readings were recorded, and if there was a difference of more than 10 mmHg, a third reading was recorded. Systolic blood pressure (SBP) ≥ 140 mmHg and/or diastolic blood pressure (DBP) reading of ≥90 mmHg were categorized as hypertension. Fasting serum triglyceride concentration ≥ 200 mg/dl was categorized as hypertriglyceridemia.

### 2.4. Anthropometric Measurements and Biochemical Parameters

Standard techniques were followed to measure the age, height, and weight of the study subjects. Medical history was obtained from all the participants, including details of their occupation, severity and duration of the disease, treatment protocol that was followed, complications encountered, and addiction, if any. Body mass index (BMI) of the study subjects was calculated. Venous blood was collected from the median cubital vein after an overnight fast of 12 hours. The blood samples were collected in sterile containers, centrifuged at 3000 rpm; the serum/plasma was separated and stored at -80°C. The enzymatic colorimetric technique based on the glucose oxidase-peroxidase method was used to measure the glucose level. All the biochemical parameters were measured using a Hitachi-912 Autoanalyser (Hitachi, Mannheim, Germany). Plasma visfatin levels were estimated using an ELISA Kit (Thermo Scientific, USA).

### 2.5. Profiling of Inflammatory Cytokines Using Multiplex Assay

The levels of inflammatory cytokines such as proinflammatory cytokines, including TNF-*α*, IL-1*β*, IL-6, IL-17A, and IL-17F in the plasma of the study subjects, were measured using a multiplex bead-based assay (Bio-Rad, CA, USA). Briefly, plasma samples (50 *μ*L) were taken into a Bio-Plex plate, and the assay was carried out in duplicate according to the manufacturer's instructions. The cytokine levels were measured from standard curves and expressed as pg/mL. The intra- and interassay coefficients of variation were found as less than 5%.

### 2.6. Statistical Analysis

Student's *t*-test and chi-squared test were adopted to compare quantitative and categorical parameters, respectively. The Mann-Whitney *U* test was used for non-normally distributed parameters to compare medians. Pearson's correlation tests were used to examine the association of plasma cytokine levels with clinical parameters. The Kruskal-Wallis test was adopted for multiple parameters which do not exhibit normal distribution. Multiple comparisons were corrected using Holm's correction [21]. The analysis was done using the SPSS statistical package (version 20.0; SPSS, Chicago, IL), and *p* values less than 0.05 were considered significant.

## 3. Results

### 3.1. Clinical and Biochemical Parameters of the Study Subjects

Table 1 depicts the clinical characteristics and biochemical parameters of the study subjects. The age difference was not significant among or between the hypertensive subjects, though BMI was significantly elevated in all the hypertensive subjects (groups 2 and 3) as compared to the control (group 1), there was no significant difference in the age between the hypertensive subjects, but they were comparatively older than the control subjects. There is no significant difference in the fasting plasma glucose in the study subjects. Total cholesterol was found to be elevated in group 3 as compared to group 2 (hypertension) and group 1 (normotensive) subjects. Serum triglycerides and LDL cholesterol were significantly increased in hypertensive hypertriglyceridemic subjects (group 3) compared to the other groups (groups 1 and 2).

### 3.2. Plasma Visfatin levels among the Study Subjects

Figure 1 shows the plasma levels of visfatin in the study subjects. Plasma visfatin levels were significantly elevated in hypertensive subjects (groups 2 and 3) as compared to the control (group 1) (*p* < 0.001). When visfatin levels of hypertensive subjects (group 2) were compared with hypertensive hypertriglyceridemic subjects (group3), their levels were further elevated (*p* < 0.05).

### 3.3. Levels of Proinflammatory Cytokine among the Study Subjects

Figure 2 displays proinflammatory cytokine levels in the circulation of the study subjects. All the tested proinflammatory cytokines, including TNF*-α*, IL-1*β*, IL-6, IL-17A, and IL-17F, were significantly increased in hypertensive subjects (group 2) as compared to the control (group 1). Among the tested cytokines, IL-1*β*, IL-6, IL-17A, and IL-17F were further increased in hypertensive hypertriglyceridemic subjects (group 3) compared to the hypertensive subjects (group 2). The major cytokine TNF*-α* did not show any difference between hypertensive hypertriglyceridemic subjects and hypertensive subjects.

### 3.4. Pearson's Correlation for Plasma Visfatin over Inflammatory Cytokines

Table 2 shows the Pearson correlation coefficient of plasma visfatin with inflammatory cytokines in hypertensive hypertriglyceridemic subjects (group 4). We found a positive correlation between IL-6 (*r* = 0.03; *p* = 0.360) and TNF*-α* (*r* = 0.04; *p* = 0.291).

### 3.5. Pearson's Correlation for Plasma Visfatin with Other Clinical Parameters

Table 3 shows the Pearson correlation coefficient of plasma visfatin with other clinical parameters in hypertensive hypertriglyceridemic subjects (group 4). Visfatin levels showed a positive correlation with diastolic blood pressure (*r* = 0.599; *p* = 0.009) and negative correlation with urea (*r* = −0.639; *p* = 0.01), potassium (*r* = −0.563; *p* = 0.02), and HDL cholesterol (*r* = −0.105; *p* = 0.02).

## 4. Discussion

Visfatin, a known proinflammatory cytokine, plays a significant role in many chronic inflammatory conditions, including atherosclerosis and cardiovascular diseases. Though the structure of visfatin has been unraveled, its role in hypertension, atherosclerosis, and cancer still needs to be studied thoroughly.

Our results showed significantly elevated plasma visfatin concentrations in the hypertensive subjects as compared to the control. Besides, a positive correlation was observed between plasma visfatin and diastolic blood pressure in these patients. In this context, Seo et al. have also reported enhanced plasma visfatin concentrations in women hypertensive patients with elevated diastolic blood pressure [22]. Similarly, Ingelsson et al. observed that the prevalence of hypertension corresponds with visfatin concentrations [23]. Rotkegel et al., in their study, observed markedly elevated plasma visfatin concentrations in hypertensive patients as compared to the control [24]. Moreover, in the present study, we observed no significant changes in circulating visfatin levels in normotensive subjects, showing that there is an association between circulatory visfatin and blood pressure.

Moreover, reports show that visceral obesity is associated with elevated plasma visfatin levels in hypertensive patients [25]. Our data also revealed increased BMI in hypertensive patients of all the groups as compared to the control subjects. Further, Filippatos et al. revealed that waist circumference, total cholesterol, and triglyceride levels were positively correlated with blood pressure [26]. Similarly, we observed significantly elevated serum triglycerides and LDL cholesterol concentrations in the hypertensive hypertriglyceridemic subjects compared to the other two hypertensive subjects (groups 2 and 3). Synchronous results were also obtained by Sun et al., who reported a positive correlation between visfatin and triglycerides in the serum [27].

The high levels of visfatin in the plasma of hypertensive subjects could be explained by suggesting that visfatin and blood pressure are inversely related and that adipose tissue may play a protective role in blood pressure regulation by secreting visfatin. In this regard, animal studies revealed that visfatin dose-dependently suppresses blood pressure elevation in deoxycorticosterone (DOCA) salt hypertensive rats [28].

Visfatin is a proinflammatory cytokine that is secreted by monocytes and macrophages that infiltrate tissue spaces in response to inflammation and can directly interact with vascular cells. Besides, visfatin is known to stimulate vascular smooth muscle cell (VSMC) inflammation and plays a vital role in atherosclerosis and other inflammatory diseases [29]. We observed a positive correlation between visfatin and proinflammatory cytokines such as IL-6 and TNF*-α* in hypertensive hypertriglyceridemic subjects. Similarly, Dahl et al. observed that visfatin elevated TNF-*α* and IL-8 in peripheral blood mononuclear cells *in vitro* [30]. In this context, visfatin via iNOS regulation directly affects vascular function and inflammation [31].

Earlier studies documented that visfatin acts as a growth factor and activates a few signaling pathways such as PI3K and STAT3 [32]. It has been reported that recombinant visfatin administration increases the proliferation of breast cancer MCF-7 cells [33]. Further, the elevated visfatin levels in breast cancer patients were reported to be associated with the higher development of breast cancer and worse prognosis [34, 35]. Further, the elevated visfatin increases the levels of MMPs 2 and 9, and VEGF is leading to migration, invasion, and metastasis [36].

Higher levels of visfatin in obese subjects show hypoadiponemia and hyperleptinemia, leading to obesity associated with cancer [37]. Visfatin levels influence obesity-induced adipokine involvement in the pathophysiology of cancer development [16]. In hypertensive subjects, visfatin provides a link between cancer and obesity via (i) acting as a proinflammatory cytokine linking obesity to cancer [38] and (ii) triggering the proangiogenic, invasive, and metastatic nature of visfatin in obese hypertensive subjects with hyperlipidemic conditions leading to increased estrogen levels and thereby breast cancer [39].

Thus, the synergistic increase in the levels of visfatin and the proinflammatory cytokines could play an important role in the pathogenesis of hypertension. However, visfatin is known to be linked with the activation of Akt (protein kinase B) and P 44/42 (MAPK) signaling pathways, thereby protecting the VSMC and thus the development of hypertension [40]. Moreover, Yilmaz et al. reported that visfatin plays an important role in the renin-angiotensin system [41]. Angiotensin-II is known to activate the ATI/R-JAK/STAT pathway and increase the expression of visfatin [42]. On the other hand, visfatin has been negatively correlated with circulating aldosterone [43].

Overall, the role of visfatin on inflammatory and cardiovascular diseases revealed conflicting results. Most studies showed enhanced visfatin levels in hypertension, diabetes, obesity, and renal and cardiovascular diseases. Our data correlate with the above findings. However, some studies show reduced levels of plasma visfatin, which could be due to the multifarious regulation of visfatin.

## 5. Conclusion

The outcomes of the present study have demonstrated the elevated level of plasma visfatin in hypertensive patients with hypertriglyceridemia associated with proinflammatory cytokines. Visfatin exhibits proliferative, antiapoptotic, proinflammatory, and proangiogenic properties. Moreover, circulatory visfatin was also increased in many cancers, including obesity-associated cancers, and associated with bad prognosis and higher tumor stage. Though the relationship between obesity and hypertension is well established and hypertension has been reported to be the most common comorbidity encountered in patients with cancer, visfatin may be a novel potential therapeutic target for hypertension in cancer patients and survivors.

## Figures and Tables

**Figure 1:** Serum visfatin concentrations of control and hypertensive subjects. The error bar represents the geometric mean unit with 95% confidence interval. The *p* values were calculated by Kruskal-Wallis one-way analysis of variance. *p* < 0.05 was considered significant.

**Figure 2:** Profiling of serum cytokines using a multiplex bead-based assay system between control and hypertensive subjects. The error bar represents the geometric mean unit with 95% confidence interval. The *p* values were calculated by Kruskal-Wallis one-way analysis of variance. *p* < 0.05 was considered significant.

**Table 1:** Clinical and biochemical characteristics of the study subjects.

Clinical parameters	NGT	HTN	HTN+TGL	One-way ANOVA	Brown-Forsythe test (*F* statistics)
Age (years)	43.6 ± 9.33	54.4 ± 11.2	51.9 ± 10.9	0.002	0.44
Systolic blood pressure (mm Hg)	112.0 ± 7.6	160.0 ± 19.6	164.4 ± 29.7	<0.0001	6.34
Diastolic blood pressure (mm Hg)	78.5 ± 6.7	97.3 ± 9.9	97.7 ± 5.4	<0.0001	1.27
Fasting plasma glucose (mg/dL)	95.4 ± 6.5	103.5 ± 44.5	92.4 ± 27.5	<0.0001	8.73
Urea (mg/dL)	20.6 ± 3.2	28.4 ± 5.9	25.4 ± 5.2	<0.0001	1.91
Creatinine (mg/dL)	0.8 ± 0.1	0.8 ± 0.10	0.8 ± 0.06	0.47	1.44
Sodium (mEq/L)	138.8 ± 2.8	134.1 ± 20.1	138.3 ± 1.8	0.51	0.88
Potassium (mmol/L)	4.2 ± 0.4	4.0 ± 0.8	4.1 ± 0.2	0.49	1.11
Chloride (mEq/L)	99.9 ± 3.1	100.3 ± 2.4	100.6 ± 1.6	0.82	3.21
Total serum cholesterol (mg/dL)	155.3 ± 26.1	172.0 ± 26.9	202.6 ± 27.0	<0.0001	4.74
Serum triglycerides (mg/dL)	103.2 ± 25.3	112.3 ± 27.1	238.8 ± 53.1	<0.0001	5.77
HDL cholesterol (mg/dL)	45.5 ± 6.9	46.7 ± 19.4	42.1 ± 3.3	0.64	0.49
LDL cholesterol (mg/dL)	81.8 ± 9.9	107.3 ± 26.9	112.6 ± 25.3	0.0007	8.94

All data are reported as the mean ± SD for continuous variables. *p* values were calculated using a one-way ANOVA test on PRISM software (version 6.0).

**Table 2:** Pearson correlation coefficient of proinflammatory cytokines compared with plasma levels of visfatin in HTN+TGL subjects.

Inflammatory cytokines	*r*	*p*
IL-1*β*	-0.09	0.61
IL-6	0.36^∗^	0.03
IL-17A	-0.02	0.91
IL-17F	-0.11	0.51
TNF*α*	0.29^∗^	0.04

*p* and *r* values were calculated using the Pearson correlation test at 95% confidence intervals.

**Table 3:** Pearson correlation coefficient of clinical parameters compared with plasma levels of visfatin in HTN+TGL subjects.

Clinical parameters	*r*	*p*
Age	-0.484	0.06
Systolic blood pressure	0.211	0.45
Diastolic blood pressure	0.599	0.009
Fasting plasma glucose	-0.143	0.61
Urea	-0.639	0.01
Creatinine	0.231	0.40
Sodium	0.176	0.52
Potassium	0.563	0.02
Chloride	-0.042	0.88
Total cholesterol	0.361	0.93
Triglycerides	0.308	0.26
High-density lipoprotein	-0.105	0.02
Low-density lipoprotein	0.356	0.19
Bilirubin total	0.384	0.15
Bilirubin direct	0.186	0.50

*p* and *r* values were calculated using the Pearson correlation test at 95% confidence intervals.

## Data Availability

Data is available on request.

## References

[1] James P. A., Oparil S., Carter B. L. (2014). 2014 evidence-based guideline for the management of high blood pressure in adults. *JAMA*.

[2] Muller D. N., Shagdarsuren E., Park J. K. (2002). Immunosuppressive treatment protects against angiotensin II-induced renal damage. *The American Journal of Pathology*.

[3] Mouhayar E., Salahudeen A. (2011). Hypertension in cancer patients. *Texas Heart Institute Journal*.

[4] Zhang J., Crowley S. D. (2015). Role of T lymphocytes in hypertension. *Current Opinion in Pharmacology*.

[5] Ates I., Ozkayar N., Akyel F. (2014). The relationship between asymptomatic organ damage, and serum soluble tumor necrosis factor-like weak inducer of apoptosis (sTWEAK) and interleukin-17A (IL-17A) levels in non-diabetic hypertensive patients. *BMC Nephrology*.

[6] Bautista L. E., Vera L. M., Arenas I. A., Gamarra G. (2005). Independent association between inflammatory markers (C-reactive protein, interleukin-6, and TNF-alpha) and essential hypertension. *Journal of Human Hypertension*.

[7] Guzik T. J., Hoch N. E., Brown K. A. (2007). Role of the T cell in the genesis of angiotensin II induced hypertension and vascular dysfunction. *The Journal of Experimental Medicine*.

[8] Heptinstall R. H. (1954). Renal biopsies in hypertension. *British Heart Journal*.

[9] Saddi-Rosa P., Oliveira C. S., Giuffrida F. M., Reis A. F. (2010). Visfatin, glucose metabolism and vascular disease: a review of evidence. *Diabetology & Metabolic Syndrome*.

[10] Moschen A. R., Kaser A., Enrich B. (2007). Visfatin, an adipocytokine with proinflammatory and immunomodulating properties. *Journal of Immunology*.

[11] Moschen A. R., Gerner R. R., Tilg H. (2010). Pre-B cell colony enhancing factor/NAMPT/visfatin in inflammation and obesity-related disorders. *Current Pharmaceutical Design*.

[12] Gunes F., Akbal E., Cakir E., Akyurek O., Altunbas M., Ozbek M. (2012). Visfatin may be a novel marker for identifying stages of essential hypertension in advanced age patients. *Internal Medicine*.

[13] Hajianfar H., Bahonar A., Entezari M. H., Askari G., Yazdani M. (2012). Lipid profiles and serum visfatin concentrations in patients with type II diabetes in comparison with healthy controls. *International Journal of Preventive Medicine*.

[14] Li Y., Zhang Y., Dorweiler B. (2008). Extracellular Nampt promotes macrophage survival via a nonenzymatic interleukin-6/STAT3 signaling mechanism. *The Journal of Biological Chemistry*.

[15] Otani K., Ishihara S., Yamaguchi H. (2017). Adiponectin and colorectal cancer. *Surgery Today*.

[16] Garten A., Petzold S., Korner A., Imai S., Kiess W. (2009). Nampt: linking NAD biology, metabolism and cancer. *Trends in Endocrinology and Metabolism: TEM*.

[17] Cymbaluk-Ploska A., Chudecka-Glaz A., Pius-Sadowska E., Sompolska-Rzechula A., Machalinski B., Menkiszak J. (2018). Circulating serum level of visfatin in patients with endometrial cancer. *BioMed Research International*.

[18] Sun Y., Zhu S., Wu Z. (2017). Elevated serum visfatin levels are associated with poor prognosis of hepatocellular carcinoma. *Oncotarget*.

[19] Mohammadi M., Mianabadi F., Mehrad-Majd H. (2019). Circulating visfatin levels and cancers risk: a systematic review and meta-analysis. *Journal of Cellular Physiology*.

[20] Monteiro R., Azevedo I. (2010). Chronic inflammation in obesity and the metabolic syndrome. *Mediators of Inflammation*.

[21] Aickin M., Gensler H. (1996). Adjusting for multiple testing when reporting research results: the Bonferroni vs Holm methods. *American Journal of Public Health*.

[22] Seo J. A., Jang E. S., Kim B. G. (2008). Plasma visfatin levels are positively associated with circulating interleukin-6 in apparently healthy Korean women. *Diabetes Research and Clinical Practice*.

[23] Ingelsson E., Larson M. G., Fox C. S. (2007). Clinical correlates of circulating visfatin levels in a community-based sample. *Diabetes Care*.

[24] Rotkegel S., Chudek J., Spiechowicz-Zaton U., Ficek R., Adamczak M., Wiecek A. (2013). The effect of sodium restricted diet on plasma visfatin levels in hypertensive patients with visceral obesity. *Kidney & Blood Pressure Research*.

[25] Dogru T., Sonmez A., Tasci I. (2007). Plasma visfatin levels in young male patients with uncomplicated and newly diagnosed hypertension. *Journal of Human Hypertension*.

[26] Filippatos T. D., Derdemezis C. S., Gazi I. F. (2008). Increased plasma visfatin levels in subjects with the metabolic syndrome. *European Journal of Clinical Investigation*.

[27] Sun G., Bishop J., Khalili S. (2007). Serum visfatin concentrations are positively correlated with serum triacylglycerols and down-regulated by overfeeding in healthy young men. *The American Journal of Clinical Nutrition*.

[28] Rezk M. Y. (2014). Visfatin and cardiovascular protection. *Journal of Drug Delivery and Therapeutics*.

[29] Hognogi L. D. M., Simiti L. V. (2016). The cardiovascular impact of visfatin - an inflammation predictor biomarker in metabolic syndrome. *Clujul Medical*.

[30] Dahl T. B., Yndestad A., Skjelland M. (2007). Increased expression of visfatin in macrophages of human unstable carotid and coronary atherosclerosis. *Circulation*.

[31] Romacho T., Azcutia V., Vazquez-Bella M. (2009). Extracellular PBEF/NAMPT/visfatin activates proinflammatory signalling in human vascular smooth muscle cells through nicotinamide phosphoribosyltransferase activity. *Diabetologia*.

[32] Al-Suhaimi E. A., Shehzad A. (2013). Leptin, resistin and visfatin: the missing link between endocrine metabolic disorders and immunity. *European Journal of Medical Research*.

[33] Kim J. G., Kim E. O., Jeong B. R. (2010). Visfatin stimulates proliferation of MCF-7 human breast cancer cells. *Molecules and Cells*.

[34] Lee Y. C., Yang Y. H., Su J. H., Chang H. L., Hou M. F., Yuan S. S. (2011). High visfatin expression in breast cancer tissue is associated with poor survival. *Cancer Epidemiology, Biomarkers & Prevention*.

[35] Dalamaga M., Diakopoulos K. N., Mantzoros C. S. (2012). The role of adiponectin in cancer: a review of current evidence. *Endocrine Reviews*.

[36] Lin T. C. (2019). The role of visfatin in cancer proliferation, angiogenesis, metastasis, drug resistance and clinical prognosis. *Cancer Management and Research*.

[37] Gui Y., Pan Q., Chen X., Xu S., Luo X., Chen L. (2017). The association between obesity related adipokines and risk of breast cancer: a meta-analysis. *Oncotarget*.

[38] Jarde T., Perrier S., Vasson M. P., Caldefie-Chezet F. (2011). Molecular mechanisms of leptin and adiponectin in breast cancer. *European Journal of Cancer*.

[39] Assiri A. M. A., Kamel H. F., Hassanien M. F. (2015). Resistin, visfatin, adiponectin, and leptin: risk of breast cancer in pre- and postmenopausal saudi females and their possible diagnostic and predictive implications as novel biomarkers. *Disease Markers*.

[40] Hausenloy D. J., Yellon D. M. (2009). Cardioprotective growth factors. *Cardiovascular Research*.

[41] Yilmaz M. I., Saglam M., Carrero J. J. (2008). Serum visfatin concentration and endothelial dysfunction in chronic kidney disease. *Nephrology, Dialysis, Transplantation*.

[42] Chang L., Yang R., Wang M. (2012). Angiotensin II type-1 receptor-JAK/STAT pathway mediates the induction of visfatin in angiotensin II-induced cardiomyocyte hypertrophy. *The American Journal of the Medical Sciences*.

[43] Takebayashi K., Suetsugu M., Wakabayashi S., Aso Y., Inukai T. (2007). Association between plasma visfatin and vascular endothelial function in patients with type 2 diabetes mellitus. *Metabolism: Clinical and Experimental*.

